# Deep Learning and Improved HMM Training Algorithm and Its Analysis in Facial Expression Recognition of Sports Athletes

This article has been retracted.

**DOI:** 10.1155/2022/1027735

**Published:** 2022-01-18

**Authors:** Shaolong Li, Yijun Bai

**Affiliations:** ^1^Sports Reform and Development Research Center, Institute of Physical Education, Henan University, Kaifeng 475001, Henan, China; ^2^Guangdong Tianhe Branch of China Telecom, Guangzhou 510632, Guangdong, China

## Abstract

Facial expressions are an auxiliary embodiment of information conveyed in the communication between people. Facial expressions can not only convey the semantic information that people want to express but also convey the emotional state of the speaker at the same time. But for sports athletes in training and competitions, it is usually not convenient to communicate directly. This paper is based on deep learning and an improved HMM training algorithm to study the facial expression recognition of sports athletes. It proposes the construction of deep learning of multilayer neural network, and the rank algorithm is introduced to carry out face recognition experiments with traditional HMM and class-specific HMM methods. The experimental results show that, with the increase of rank value, the class-specific recognition rate is up to 90%, the detection rate is 98% and the time-consuming is 2.5 min, which is better than HMM overall.

## 1. Introduction

### 1.1. Background

In recent years, the domestic sports industry has developed in an all-round way, and the level has always been at the forefront of the world. Chinese athletes have made great contributions to this. However, in the conduct of specific events, it is often impossible to meet the needs and indications of our athletes. We need to use some algorithms to capture the facial expressions of sports athletes for recognition and analysis. The history of computer vision technology can be traced back more than 70 years ago when it was mainly used in the field of pattern recognition. It mainly used some computer equipment to imitate the visual mechanism of living beings to process the information contained in the image. Humanized operation, the main purpose of studying computer vision, is to let computers replace humans to do some tedious tasks and reduce the burden of human work. Up to now, with the continuous improvement of graphics processor performance, deep learning technology has been successfully applied in the field of computer vision, and computers can completely replace or even surpass humans in certain image processing tasks.

### 1.2. Significance

In real life, human beings mainly obtain all things and information around them through vision. Facial expression recognition technology is now relatively mature, and it is an important research discipline in the field of computer vision. At the same time, the research on the facial expression recognition of sports athletes using deep learning and improved HMM training algorithm has an important impact on the performance of sports athletes.

### 1.3. Related Work

Because performance expectations play an important role in the success of technical sports in football and martial arts, there is evidence that famous athletes who play in public are performing well in terms of transfer expectations. There are few studies on whether martial arts and emotional outbursts affect athletic performance expectations. Shih's study compares the expected performance of multiple athletes and is consistent with the function of emotional identification. Preliminary research has found that normal performance expectations do not depend on strong practice data. The expected performance of Taekwondo athletes is related to the function of emotional identification, while the expected function of weight loss is not related to the function of emotional identification. Research shows that, in competitive sports such as Taekwondo, emotional identification plays an important role in predicting behavior, but the range of practicality is too small [1]. Research shows that MNS is directly related to the development of social science. This social awareness is directly affected by facial recognition skills. Therefore, the mechanism of MNS can be used to establish contact with face recognition. In the process of recognizing facial expressions, mirror neurons stimulate and provide internal simulations of observed motor behaviors, thus triggering such emotional disturbances in the observer's heart. This phenomenon is called motor coordination. This kind of motion resonance can recognize the emotions, feelings, states, or actions that are perceived. Jouini studied the influence of the sports expertise and effort intensity between karate players (KD) and football players (SC) on the facial fatigue recognition of opponents. He assumed that long-term combat sports training could positively affect the opponent's facial expression processing ability. The results show that the motion resonance increases with the increase of exertion intensity. In short, research shows that long-term karate practice can ensure the development of the strength of the opponent's facial expression, which has certain enlightenment for our research [2]. In-depth learning is a branch of engineering that seeks to model high-level data extraction using multiple layers of neurons with complex structures or nonlinear modifications. With the increase in data size and computing power, virtual networks with more complex features have gained widespread attention and have been used in many fields. Hao conducts in-depth training in neural networks, including popular architectural models and training algorithms, but the research content is not deep enough [3]. In-depth learning algorithms, especially convergence networks, have quickly become the preferred method for analyzing medical imaging. Through the research of deep learning technology in the construction of an artificial neural network, this paper has some inspiration. Litjens reviewed the first in-depth training tips related to medical imaging analysis and collected more than 300 streams in this area, most of which appeared last year. At the same time, it explores the use of in-depth learning in image isolation, object search, segregation, recording, and other activities and provides a brief overview of the study in each area, discussing open-ended challenges and guidelines for day-to-day research, but the use of procedures is too complicated [4]. Separation is one of the most popular topics in hyperspectral vision. Chen introduces an in-depth study of hyperspectral data analysis for the first time. First, the applicability of the stacked autoencoder is verified according to the classic classification method based on spectral information. Secondly, a classification method based on spatial dominance information is proposed. He then proposed a new depth training system to combine these two features, from which you could get a higher degree of accuracy. The process is a combination of primary component analysis (PCA), in-depth learning architecture, and material regression. Essentially, like in-depth training architecture, automated encoders are designed to record practical improvements. Experimental results on widely used hyperspectral data show that the classifier integrated into this in-depth learning process performs well. In addition, the proposed deep neural network opens a new window for future research, highlighting the great potential of training-based methods in the proportion of hyperspectral data, but it has not yet been reused [5]. The Markov Custom Parameter Estimation Method (HMM) is easy to get into the best area and has the highest requirements on the main bases, which can also lead to a merge event. In order to improve the power and recognition function of the model, Li proposed a new HMM algorithm IPSAA. Firstly, in particle swarm optimization (PSO), the parameters such as the incentive factor in the ant colony algorithm (ACA) are adaptively improved. Secondly, the fitness function value of the particle historical optimal solution is used after the coarse search of the particle swarm algorithm to adjust the initial pheromone distribution in the fine search of the ant colony algorithm. Finally, the Baum–Welch (B–W) algorithm is used to improve the region in the forthcoming global solution. The new algorithm not only solves the problem of BW dependence on the initial value and falling in the optimal range but also makes full use of the universal IPS search feature but is not useful [6].

### 1.4. Innovation

This paper mainly studies and improves the training algorithm of deep learning HMM. The innovations are as follows: (1) Improved algorithm: analyze the application of HMM in facial recognition and its algorithm theory, and propose an improved HMM training algorithm by studying the principles and shortcomings of HMM. The class-specific HMM method obtains a better way by retaining the information of the given maximum dimension. It assigns an independent feature system to each class. (2) Without the estimation error of probability density function, even without sufficient feature statistics, the optimal classifier can be established by class-specific sufficient statistics. (3) Facial expression recognition comparison experiment: based on the facial expression data of 50 people, a small database is built for training and recognition. The traditional HMM algorithm and the improved class-specific HMM training algorithm are, respectively, applied to train the database, and the superiority of the improved class-specific HMM is verified by performing facial expression recognition experiments on the two sets of parameters and comparing the recognition rates.

## 2. Deep Learning and Improved HMM Training Algorithm

### 2.1. Deep Learning Technology

The core content of deep learning is to build artificial neural networks and through continuous training of large amounts of data to meet certain specific needs. The idea of deep learning is to extract the information contained in the input hierarchically by constructing a multilayer neural network; the construction of a multilayer neural network refers to the introduction of hidden layers between the input layer and the output layer of the single computing layer perceptron as the internal representation of the “input mode,” so that the single computing layer perceptron becomes a multi (computing)-layer perceptron, and the neurons between adjacent layers are connected to each other [7]. Deep learning can be understood in two parts: one is depth, which is to build a multilayer network to achieve the purpose of depth; the other is learning, using a certain algorithm to update the parameters of each layer until convergence. Deep learning is a supervised learning method. In the learning process, the labels of the training samples and the objectives to be achieved need to be given, and the network parameters of each layer are continuously adjusted to optimize the network performance of deep learning.

The most critical technology of deep learning is how to train and build a good neural network. This section will introduce several key technologies for training neural networks: backpropagation and gradient descent [8].

#### 2.1.1. Backpropagation

The deep learning training algorithm was officially established because of the backpropagation algorithm. It is the most common and effective method to update the network parameters of each layer. The specific process is as follows: first, the training set is forwarded through the neural network, and at the end, one layer gets the output value of the network, then calculates the difference between it and the true value, and propagates the error layer by layer from the last layer to the input layer. In the process of propagating errors, the parameters of this layer can be based on the previous layer, the propagated error is adjusted, and this process is repeated until the error converges to the minimum [9].

#### 2.1.2. Gradient Descent

The error of each layer in the artificial neural network can be obtained through the backpropagation algorithm. According to the error of each layer, the update gradient of the parameters of this layer can be calculated, and then the parameters of each layer can be updated using the descent method. The gradient descent algorithm will be introduced here. How does it work? The direction of the gradient refers to the direction of the maximum directional derivative of the function at a certain point [10]. Generally, the closer the target value, the smaller the step length and the slower the progress. The gradient descent method cannot be used to find the optimal value in all cases. When the curve of the objective function is convex, the gradient descent method can be used to find the global optimal solution, but in general, the objective function is not strictly convex. The solution obtained by the gradient descent method is the local optimal solution. Common gradient descent methods include stochastic gradient descent and batch gradient descent. The main difference between the two methods is the difference in the calculation of the gradient [11].

The classic neural networks include the following.

*(1) Convolutional Neural Network*. Inspired by the principle of animal visual perception, researchers proposed the convolutional neural network (CNN). The convolution layer is the core network layer in CNN, which is composed of several convolution units. A variety of features are extracted through convolution nuclear energy with different shapes. A low-level convolution layer usually extracts some low-level features, such as color, texture, and brightness. Higher-level networks can extract low-level feature combinations into complex high-level features, and the face embedding process is output by training the convolutional neural network [12]. The activation layer adds nonlinear transformation to the network through the activation function to strengthen the expression ability of the network to the input. The full connection layer usually converts the two-dimensional feature map into a one-dimensional feature vector for classification [13].  Figure 1 is a process diagram from the full connection layer to the classifier layer.

*(2) Recurrent Neural Network*. The earliest neural network-based language model was proposed by Bengio. Later, in 2010, Mikolov improved the model proposed by Bengio and proposed a recurrent neural network model RNN (Recurrent Neuron Network). RNN has a special structure, LSTM (Long Short-Term Memory), which has recently been improved and promoted by researchers, and has achieved great success [14]. With the vigorous development of the field of artificial intelligence, RNN has begun to quickly find a large number of applications in natural language processing, speech recognition, and other fields. Compared with other networks, RNN can process sequence data, and its biggest difference from convolutional neural networks is that the hidden layers are connected to each other. In RNN, the output of the current network layer is related to the output of the previous network layer. It will memorize the information of the previous network layer and affect the output of the current network layer. Ideally, RNN can process sequence data of any length, but in reality, the current state of the data is only related to the state of the first few data, so it is not necessary to pay attention to all the data in the sequence [15].

### 2.2. HMM Training Algorithm

HMM stands for Hidden Markov Model, which is a probability model established and developed on the basis of the Markov chain to describe statistical characteristics. Since the state of the event cannot be seen intuitively, it can only be perceived by the observed value, so it is called HMM [16]. The HMM training method is essentially a gradient descent method, and it is possible to reach a local minimum during the training process. Therefore, the selection of the initial value is more important. A good initial value can avoid the problem of local minima. The initial value can be selected by adding certain optimization methods.

Since the state of HMM cannot be directly observed, it needs to be reflected indirectly through an observation vector, and the distribution of each state is also random, so HMM can be seen as a double random process. Among them, the randomly generated sequence is called the state sequence, and the sequence composed of the observations generated by each state is called the observation sequence [17]. According to these parameters, the probability of a certain event occurring at any time can be calculated. The specific HMM form is defined as follows.

Let *A* denote the set consisting of *N* possible states, *B* denote the set consisting of *M* possible observations, and *q*_*t*_ denote the state at *t*; obviously, *q*_*t*_ ∈ *A*.

(1) $$\begin{array}{c} A=\left\{A_{1},A_{2},\ldots ,A_{N}\right\},\\ B=\left\{B_{1},B_{2},\ldots ,B_{N}\right\}. \end{array}$$

(1) *L* represents a set of observation sequences, *K* represents the state sequence corresponding to *L*, and its length is *l*.
  (2) $$\begin{array}{c} L=\left(l_{1},l_{2},\ldots ,l_{b}\right),\\ K=\left(k_{1},k_{2},\ldots ,k_{b}\right). \end{array}$$
Normally, a frontal face image contains five prominent parts of the forehead, eyes, nose, mouth, and chin in sequence. Even if the head is deflected or tilted to a certain extent, their order will not change [18].  Figure 2 shows how the observation sequence is generated.
(2) State transition probability matrix *S*={*s*_*ij*_},
  (3) $$\begin{array}{c} s_{ij}=P\left(q_{t+1}=A_{j}|q_{t}=A_{i}\right),\;1\leq i,j\leq N, \end{array}$$
represents the probability of state *S*_*i*_ was transitioning to *S*_*j*_ from time *t* to *t* + 1.
(3) Observation probability matrix *T*={*t*_*j*_(*k*)},
  (4) $$\begin{array}{c} T=\left\{t_{j}\left(o_{t}=V_{k}|q_{t}=A_{j}\right)\right\},\;1\leq j\leq N;1\leq k\leq M, \end{array}$$
indicates the probability of generating was a certain observation value at time *t*.
(4) The initial probability vector *π*={*π*_*i*_},
  (5) $$\begin{array}{c} \pi_{i}=P\left(q_{1}=A_{i}\right),\;1\leq i\leq N, \end{array}$$
represents the probability of state *A*_*i*_ at *t* = 1.

Therefore, the entire HMM can be expressed as

(6) $$\begin{array}{c} \lambda =\left(\pi ,S,T\right). \end{array}$$

In fact, HMM consists of two parts. The first part is a Markov chain, which is described by *π* and *S*, and the second part is a random process, which is described by *T*.  Figure 3 is a schematic diagram of the structure of the HMM.

Given the initial model of *λ*=(*π*, *S*, *T*) and the sequence of observations *L*=(*l*_1_, *l*_2_,…, *l*_*b*_),

1. Solve the probability problem [19]: assuming *λ*=(*π*, *S*, *T*) and *L*=(*l*_1_, *l*_2_,…, *l*_*b*_), calculate the probability *P*(*L|λ*). This problem can be seen as a matching problem between the model and the sequence of observations, and it is solved by the forward-backward algorithm.
2. Parameter estimation problem [20]: assuming *λ*=(*π*, *S*, *T*) and *L*=(*l*_1_, *l*_2_,…, *l*_*b*_), use the maximum likelihood estimation method to calculate the model parameters *λ*=(*π*, *S*, *T*), so that the probability of generating a certain observation sequence *P*(*L|λ*) reaches the maximum. This problem was created to help us do our best to optimize parameters and solve the generated set of observations and was solved by the Baum–Welch algorithm.
3. Prediction problem: given *λ*=(*π*, *S*, *T*) and *L*=(*l*_1_, *l*_2_,…, *l*_*b*_), find the state sequence *K*=*k*_1_, *k*_2_,…, *k*_*b*_ when the conditional probability *C* of the observation sequence is maximized. This problem is to reveal the deep meaning of HMM, and often such a state sequence is realized through the optimization of the Viterbi algorithm [21].  Figure 4 shows the relationship between the three basic issues of HMM.

Firstly, the parameters of *λ*=(*π*, *S*, *T*) and *L*=(*l*_1_, *l*_2_,…, *l*_*b*_) are optimized by the Baum–Welch algorithm, the model matching problem is solved by a forward-backward algorithm, and the optimal state sequence is found by the optimization of the Viterbi algorithm.

Given the model and observation sequence, when solving the probability problem, the most direct method is to solve it according to the probability calculation formula; in this regard, we introduce the forward-backward algorithm. The forward-backward algorithm is relatively simple and stable in the face of data with a large amount of calculation, and it is easy to find the local optimal value [22, 23].

#### 2.2.1. Forward Algorithm

Given model *λ*, at time *t*, the observation sequence is *L*=(*l*_1_, *l*_2_,…, *l*_*b*_). When the state is *A*_*i*_, define *α*_*i*_(*t*) as the forward probability, and the observation sequence probability *P*(*L|λ*) can be obtained recursively, denoted as

(7) $$\begin{array}{c} \alpha_{i}\left(t\right)=P\left(l_{1},l_{2},\ldots ,l_{b},q_{t}=A_{i}|\lambda \right),\\ c_{i}\left(l_{t+1}\right)={c_{i}\left(k\right)|}_{l_{t+1}=B_{k}}. \end{array}$$

This kind of algorithm needs to calculate *N*(*N* + 1)(*T* − 1) + *N* times of multiplications so that the amount of calculation is directly reduced from the order of *TN*^*T*^ to *N*^2^*T*, which greatly reduces the computational complexity.

#### 2.2.2. Backward Algorithm

Similarly, given the HMM model *λ*, when the state is *A*_*i*_ at time *t*, the probability that the observation sequence from *t* + 1 to *T* is *l*_*t*+1_, *l*_*t*+2_,…, *l*_*b*_ is defined as the backward probability, denoted as

(8) $$\begin{array}{c} \beta_{i}\left(t\right)=P\left(l_{t+1},l_{t+1},\ldots ,l_{b},q_{t}=A_{i}|\lambda \right). \end{array}$$

The forward-backward algorithm can simplify the calculation when solving *P*(*L|λ*), and the calculation amount *N*^2^*T* is also an order of magnitude. The formula can usually be written uniformly as

(9) $$\begin{array}{c} P\left(L|\lambda \right)=\sum_{i=1}^{N}\sum_{j=1}^{N}\alpha_{i}\left(i\right)x_{ij}c_{j}\left(l_{t+1}\right)\beta_{t+1}\left(j\right),\;1\leq t\leq T-1. \end{array}$$

In fact, the parameter estimation problem mainly describes the training process of the model. Through parameter training, *P*(*L|λ*) is maximized, and the Baum–Welch algorithm is generally used to solve it. Given model *λ* and observation sequence *L*, let *p*_*t*_(*i*) be the probability of being in state *A*_*i*_ at time *t* and satisfy ∑_*i*=1_^*N*^*p*_*t*_(*i*)=1. Then, there are

(10) $$\begin{array}{c} p_{t}\left(i\right)=P\left(q_{t}=A_{i}|L,\lambda \right). \end{array}$$

The probability of passing forward and backward is defined as

(11) $$\begin{array}{c} \alpha_{t}\left(i\right)\beta_{t}\left(i\right)=P\left(q_{t}=A_{i},L|\lambda \right). \end{array}$$

So,

(12) $$\begin{array}{c} p_{t}\left(i\right)=\frac{P\left(q_{t}=A_{i},L|\lambda \right)}{P\left(L|\lambda \right)}=\frac{\alpha_{t}\left(i\right)\beta_{t}\left(i\right)}{P\left(L|\lambda \right)}=\frac{\alpha_{t}\left(i\right)\beta_{t}\left(i\right)}{\sum_{j=1}^{N}\alpha_{t}\left(i\right)\beta_{t}\left(i\right)}. \end{array}$$

Let *κ*_*t*_(*i*, *j*) be the probability of being in state *A*_*i*_ at time *t* and being in *A*_*j*_ at time *t* + 1; then,

(13) $$\begin{array}{c} \kappa_{t}\left(i,j\right)=P\left(q_{t}=S_{i},q_{t+1}=S_{j}|L,\lambda \right). \end{array}$$

The probability calculation formula can be obtained:

(14) $$\begin{array}{c} \kappa_{t}\left(i,j\right)=\frac{P\left(q_{t}=A_{i},q_{t+1}=A_{j},L|\lambda \right)}{P\left(L,\lambda \right)}=\frac{P\left(q_{t}=A_{i},q_{t+1}=A_{j},L|\lambda \right)}{\sum_{i=1}^{N}\sum_{j=1}^{N}\alpha_{t}\left(i\right)x_{ij}c_{j}\left(l_{t+1}\right)\beta_{t+1}\left(j\right)}. \end{array}$$

Figure 5 is the principle of the Baum–Welch algorithm.

After defining the evaluation method, the forward probability *α*_*t*_(*i*) and backward probability *β*_*t*+1_(*j*) of the visible state chain are maximized, the initialization model parameters are optimized, and the iteration is repeated continuously.

The parameter learning and estimation of HMM can be realized by the EM algorithm, and the specific process is as follows:

*(1) Determine the Log-Likelihood Function*. Since the HMM model contains an implicit observation sequence *L*, the model and its log-likelihood function can be expressed as

(15) $$\begin{array}{c} P\left(L|\lambda \right)=\sum_{K}P\left(L|K,\lambda \right)P\left(K|\lambda \right), \end{array}$$

(16) $$\begin{array}{c} Y\left(\lambda ,\bar{\lambda }\right)=\sum_{K}\log\;P\left(L,K|\lambda \right)P\left(L,K|\bar{\lambda }\right). \end{array}$$

Here, *λ* is the HMM parameter that needs to be calculated, and $\bar{\lambda }$ is its current estimated value also because

(17) $$\begin{array}{c} P\left(L,K|\lambda \right)=\pi_{q_{1}}c_{q_{1}}\left(l_{1}\right)x_{q_{1}q_{2}}c_{q_{2}}\left(l_{2}\right),\ldots ,x_{q_{T-1}q_{T}}c_{q_{T}}\left(l_{T}\right). \end{array}$$

Therefore, formula (16) can be written as

(18) $$\begin{array}{c} Y\left(\lambda ,\bar{\lambda }\right)=\underset{K}{\sum }\log\;\pi_{q_{1}}P\left(L,K|\bar{\lambda }\right)+\underset{K}{\sum }\left(\overset{T-1}{\underset{t=1}{\sum }}\log\;x_{q_{1}q_{2}}\right)P\left(L,K|\bar{\lambda }\right)+\sum_{K}\left(\overset{T}{\underset{t=1}{\sum }}\log\;c_{q_{t}}\left(l_{t}\right)\right)P\left(L,K|\bar{\lambda }\right). \end{array}$$

*(2) Calculate Model Parameters*. Taking the maximum value of $\sum_{K}\log\;\pi_{q_{1}}P\left(L,K|\bar{\lambda }\right)$ as an example, it can be written as

(19) $$\begin{array}{c} \sum_{K}\log\;\pi_{q_{1}}P\left(L,K|\bar{\lambda }\right)=\sum_{i=1}^{N}\log\;\pi_{i}P\left(L,q_{1}=i|\bar{\lambda }\right). \end{array}$$

### 2.3. Evaluation of Facial Expression Recognition

When a sports athlete is in a competition, how to capture and lock the target person's face from a complex environment and recognize and analyze his facial expression is an important problem. For a dynamic target, let the computer complete the automatic identification; the accuracy must be guaranteed. At the same time, the influence of the external environment must be taken into consideration, such as the change of the brightness of the light, the positioning of the target person, the rapid change of expression, the similarity of some facial expressions, and the lack of samples in the model library, all of which need to be broken through one by one.

The data set is an important part of facial expressions and one of the key points for obtaining a good facial expression model. The rapid development of facial expression recognition is inseparable from the accumulation and use of effective data. Google's FaceNet has trained a highly accurate model with 200 million massive data. Many research teams have produced information-rich, high-quality public data sets. The following will introduce some commonly used public data sets with a large amount of data. The data sets can be divided into two categories. One is the public data set that is generally used for training. The other is the public data set used to test the accuracy of the evaluation model. Some brief information of all data sets is listed in Table 1.

In order to more accurately recognize the facial expressions of sports athletes, we have introduced class-specific HMM algorithms for improvement. Class-specific methods can retain as much information as possible by reducing the dimension, and increasing the dimension can obtain better probability density function estimation, so an appropriate value needs to be taken between the two, and a better way is obtained by retaining the information of the given maximum number of dimensions. It classifies and adapts to the changes of ambient light, the positioning of target characters, expression changes, and so on and assigns an independent feature system to each class. At the same time, a large number of athletes' facial expression data are collected to solve the problems of similarity of some facial expressions and lack of samples in the model database. When the state of each Hidden Markov Model has sufficient statistical information, the class-specific method can be extended to the HMM modeling problem. Unlike the likelihood function in the traditional HMM, the class-specific HMM uses class-specific statistics to define the likelihood function. Under certain conditions (when there is only noise, the probability of *x* is 1), the maximum value of the maximum likelihood function of the class-specific HMM is equal to the maximum value of the traditional model. Even if there are no sufficient feature statistics, the optimal classifier can still be established from the class-specific sufficient statistics. Because the class-specific Baum–Welch algorithm maximizes the real likelihood function, the sufficiency of the feature system does not constitute a theoretical problem.

The class-specific HMM algorithm uses a different feature set and defines a probability density function for the observation value of each state. Parameter estimation for the standard parameters of the input data space: if the state-dependent feature set has enough statistical information to distinguish each independent state, then the best classifier can be obtained.

First, the local neighborhood and global prior saliency map of all superpixels in facial expressions are used as the input of a convolutional neural network, the local context saliency map is calculated, and then it is combined with the local neighborhood of all superpixels on the depth image. As the input of another convolutional neural network, the initial saliency map is obtained [24]. After further optimization by the optimization method in this chapter, the final saliency map is obtained.  Figure 6 shows the overall flowchart.

The so-called training is to determine a set of optimized HMM parameters for each athlete. Each model can use single or multiple images for training, then establish an initial model, and use the Baum–Welch algorithm to reevaluate each parameter. Continuously adjust the model to obtain a new model until an HMM model that best characterizes the facial expressions of sports athletes is obtained. Recognition is the process of capturing the facial expression of the target person to find the best match based on the established facial expression model library.

## 3. Deep Learning and Improved HMM Training Algorithm and Its Experiment in Facial Expression Recognition of Sports Athletes

In order to evaluate the algorithm, the concepts of verification probability (hit rate) and false alarm rate are introduced. In the verification model, a person's facial expression *x* claims to be the person's *y* image, and the system accepts or rejects this claim (if the *x*, *y* image belongs to the person, it is recorded as *x*∼*y*; otherwise, it is recorded as *x* ≠ *y*). In the formal case, when *x*∼*y* is correct, the algorithm accepts the probability of *x*∼*y*. This is called the verification probability, denoted by *P*_*a*_. The second is the probability of false verification acceptance. When *x* ≠ *y*, the algorithm accepts the probability of *x*∼*y*. This is the so-called false alarm rate, represented by *P*_*b*_. When the training set is *Y* = {*y*}, verifying a person's identity is equivalent to a detection problem. This detection problem includes finding *x*∼*y* images in the test set *p* ∈ *P*.

For the training set and test set of a given picture set, it is basically *s*_*i*_(*k*) to judge whether the recognition is correct. This judgment is made by Neyman–Pearson observations. If *s*_*i*_(*k*) ≤ Rank confirms the assertion, it is considered that the recognition is correct; if *s*_*i*_(*k*) > Rank rejects the assertion, it is considered that the recognition is wrong. Through the Neyman–Pearson theory, the determined rule increases the verification rate for a given false alarm rate *α*.

In the experiment, we selected 50 subjects, each with 10 categories of facial expression images, and a total of 500 facial expression images formed a small database. The 10 types of facial expressions are divided into smiles, wink gestures, close eyes, laughs, and serious. Among them, there are 4 types of images with similar expressions, which are used to test the capture accuracy and recognition accuracy of the algorithm. The facial features of different ages are very different, and there will be different recognition rates in facial recognition. At the same time, in order to verify the feasibility and superiority of the improved class-specific HMM algorithm for facial expression recognition, the traditional HMM algorithm will be used for comparison. The number of people in 4 types of similar facial expression experiments is shown in Table 2. The distribution of the remaining 6 types of facial expression experiment population is shown in Table 3 [25, 26].

## 4. Deep Learning and Improved HMM Training Algorithm and Its Experimental Results and Analysis in Facial Expression Recognition of Sports Athletes

Figure 7 shows the accuracy of facial recognition for the six different facial expressions among male and female research subjects.

Figure 8 shows the accuracy of facial recognition for 4 kinds of similar expressions in male and female subjects.

It can be seen from Figure 8 that the two methods are still slightly different for testing facial expressions with similar expressions, except that the exact number of male calm facial expressions is the same, which is 11 people. On the whole, the class-specific HMM algorithm has a higher accuracy rate than the traditional HMM.

On a small database, take the facial expressions inside as samples for model training and use traditional HMM and class-specific HMM methods to perform face recognition experiments, respectively. As the rank value increases, the changes in the recognition rates of the six facial expressions obtained by the two algorithm experiments are shown in Figure 9.

It can be seen from Figure 9 that while the fault tolerance rate increases, the recognition rate increases; the higher the fault tolerance rate, the higher the recognition rate. In a small database, when rank = 7, the recognition rate of class-specific HMM has increased to 90%, while the recognition rate of traditional HMM has reached 95%. This shows that when rank = 7, the traditional HMM method is better than the class-specific HMM method. The recognition rate is high, and the performance is better. For traditional HMM, when rank = 10, the recognition rate is 1. For class-specific HMM facial expression recognition, when rank = 10, the recognition rate reaches 95%. On the other hand, it shows that traditional HMM has better performance and better performance than class-specific recognition.

Figure 10 is a graph showing changes in facial expression recognition rates obtained by experiments on a small database of the two algorithms for four facial recognition situations with similar facial expressions among male and female subjects as the rank value increases.

From Figure 10, it can be seen that, regardless of whether it is male or female and whether it is a class-specific HMM or HMM, the recognition rate decreases as a whole, especially when rank = 1, and the recognition rate decreases by about 10%. It shows that, in recognition of similar facial expressions, the current algorithms are not perfect enough.

Table 4 shows the detection rates of class-specific HMM and HMM methods in a small database, the total time, and the average time per sheet. The detection rate refers to the number of recognitions, regardless of whether the recognition is accurate.

It can be seen from Table 4 that the detection rates of both the class-specific HMM and HMM methods are still relatively high; especially, the class-specific HMM method is as high as 98%. In terms of time consumption, the class-specific HMM method is half less than the HMM.

## 5. Conclusions

With the continuous development of deep learning and improved HMM training methods, the measurement standards and accuracy of facial recognition are gradually improving, and facial expression recognition technology has been widely used in real life. At this stage of research technology, there is still not much to solve some of the problems faced in the process of face detection and recognition (such as serious occlusion, posture changes, and blurred data collected). In practice, when detecting and recognizing facial expressions, various situations may occur on the face, which will eventually affect the performance of detection and recognition, so the subsequent tasks are very difficult. On the basis of the existing methods, this paper has made some improvements and obtained better performance results in the facial expression data set, but this paper believes that further research is needed in the following aspects: (1) The problem of partial occlusion of human faces. In the current facial expression recognition technology, it is necessary to further explore new methods for the problem of occlusion. By introducing the expression key point alignment technology, the occluded parts of the face are detected, and the features of the unoccluded parts are learned. The design of a reasonable network model needs to be solved. (2) The problem of training data set. Based on the network framework of deep learning, a large amount of data is required as input during training, which can not only learn more robust features but also further prevent the network from overfitting. Therefore, the later use of data to expand related knowledge is more important. With more data sets, designing an improved generative confrontation network for data augmentation is the main direction. (3) The amount of calculation. With the spread of the Internet and the continuous presentation of massive data, the amount of image and video data continues to grow. Face detection and recognition are applied to industrial products for real-time face detection and recognition, so an efficient and accurate will become a long-term problem in this field.

## Figures and Tables

**Figure 1:** From full connection layer to classifier layer.

**Figure 2:** Generation method of observation sequence.

**Figure 3:** Composition diagram of HMM.

**Figure 4:** Relationship between three basic problems of HMM.

**Figure 5:** Principle of Baum–Welch algorithm.

**Figure 6:** Overall flowchart.

**Figure 7:** Male and female subjects had different facial expression recognition for six kinds of expressions.

**Figure 8:** Male and female subjects had different facial expression recognition for four kinds of expressions.

**Figure 9:** Changes in recognition rates of six facial expressions obtained from experiments of two algorithms.

**Figure 10:** Changes in recognition rates of four facial expressions obtained from experiments of two algorithms.

**Table 1:** Facial expression data set.

Data set	CelebA	VGG face	IJB-A
Number of people	12356	2532	24610
Number of pictures	300000	2600000	52163
Data set properties	It contains 5 feature points and 40 personal face attributes	Face area and identity tag	Face area and identity tag

**Table 2:** Number of similar facial expression experiments in 6 categories.

	Male		Female		Total
Age	16–22	23–40	16–22	23–40	—

Wry smile	20	10	15	5	50
Grievance	20	10	10	10	
Wink schematic	20	10	5	15	
Close eyes	15	15	5	15	
Cry bitterly	15	15	10	10	
Anger	10	20	10	10	

**Table 3:** Number of similar facial expression experiments in 4 categories.

	Male		Female		Total
Age	16–22	23–40	16–22	23–40	—

Smile	15	15	10	10	50
Laugh	15	15	10	10	
Calm	10	20	5	15	
Serious	10	20	5	15	

**Table 4:** Test indexes of two algorithms.

	Class-specific HMM	HMM
Detection proportion	98%	96%
Total time	2.5 min	5 min
Average time per	0.3 s	0.6 s

## Data Availability

No data were used to support this study.

## References

[1] Shih Y.-L., Lin C.-Y. (2016). The relationship between action anticipation and emotion recognition in athletes of open skill sports. *Cognitive Processing*.

[2] Jouini A. (2017). Physical effort and sport expertise on can modulate facial fatigue processing. *International Journal of Kinesiology and Sports Science*.

[3] Hao X., Zhang G., Ma S. (2016). Deep learning. *International Journal of Semantic Computing*.

[4] Litjens G., Kooi T., Bejnordi B. E. (2017). A survey on deep learning in medical image analysis. *Medical Image Analysis*.

[5] Chen Y., Lin Z., Xing Z., Wang G., Gu Y. (2017). Deep learning-based classification of hyperspectral data. *IEEE Journal of Selected Topics in Applied Earth Observations & Remote Sensing*.

[6] Li R., Zhao Q. S. (2017). An improved particle swarm-ant colony hybrid algorithm for HMM training. *International Journal of Wireless and Mobile Computing*.

[7] Lee J. (2020). Integration of digital twin and deep learning in cyber-physical systems: towards. *Smart Manufacturing*.

[8] Liu H., Wang W., Wang C. W. (2021). A novel research in low altitude acoustic target recognition based on HMM. *International Journal of Multimedia Data Engineering and Management*.

[9] Wu D. (2018). Online position recognition and correction method for sports athletes. *Cognitive Systems Research*.

[10] Lee S.-H., Kwon T.-D., Seok C.-H. (2017). Issues of historical recognition of athletes practicing traditional Korean sports(1): analysis of recognition level. *Korean Journal of Sports Science*.

[11] Suzuki F., Arai H. (2017). Clarification of recognition among injured athletes and their teammates. *Journal of Japan Society of Sports Industry*.

[12] Vignadelli L. Z., Ronque E. R. V., Bueno M. R. D. O., Dib L. R. P., Serassuelo Junior H. (2019). Motives for sports practice in young soccer and volleyball athletes. *Revista Brasileira de Cineantropometria e Desempenho Humano*.

[13] Liu Y., Ji Y. (2021). Target recognition of sport athletes based on deep learning and convolutional neural network. *Journal of Intelligent & Fuzzy Systems*.

[14] Léveillé E., Guay S., Blais C., Scherzer P., De Beaumont L. (2016). Sex-related differences in emotion recognition in multi-concussed athletes. *Journal of the International Neuropsychological Society*.

[15] Shen D., Wu G., Suk H.-I. (2017). Deep learning in medical image analysis. *Annual Review of Biomedical Engineering*.

[16] Wang X., Gao L., Mao S., Pandey S. (2016). CSI-based fingerprinting for indoor localization: a deep learning approach. *IEEE Transactions on Vehicular Technology*.

[17] Kermany D. S., Goldbaum M., Cai W. (2018). Identifying medical diagnoses and treatable diseases by image-based deep learning. *Cell*.

[18] Ye H., Li G. Y., Juang B. (2017). Power of deep learning for channel estimation and signal detection in OFDM systems. *IEEE Wireless Communication Letters*.

[19] Yang G., Lu Z., Yang J., Wang Y. (2019). An adaptive contourlet HMM–PCNN model of sparse representation for image denoising. *IEEE Access*.

[20] Ravi D., Wong C., Deligianni F. (2017). Deep learning for health informatics. *IEEE Journal of Biomedical and Health Informatics*.

[21] Qiao L., Dang S., Shihada B., Alouini M.-S., Nowak R., Lv Z. (2021). Can blockchain link the future?. *Digital Communications and Networks*.

[22] Zeng Y., Chen G., Li K., Zhou Y., Zhou X., Li K. (2019). M-skyline: taking sunk cost and alternative recommendation in consideration for skyline query on uncertain data. *Knowledge-Based Systems*.

[23] Lv Z. (2019). The security of internet of drones. *Computer Communications*.

[24] Yang S., Deng B., Wang J. (2019). Scalable digital neuromorphic architecture for large-scale biophysically meaningful neural network with multi-compartment neurons. *IEEE Transactions on Neural Networks and Learning Systems*.

[25] Yang B., Li X., Hou Y. (2020). Non-invasive (non-contact) measurements of human thermal physiology signals and thermal comfort/discomfort poses-a review. *Energy and Buildings*.

[26] Xie S., Yu Z., Lv Z. (2021). Multi-disease prediction based on deep learning: a survey. *Computer Modeling in Engineering & Sciences*.

